This article has been retracted.

# Unsupervised Data Mining and Effect of Fast Rehabilitation Nursing Intervention in Fracture Surgery

**DOI:** 10.1155/2022/7087844

**Published:** 2022-01-25

**Authors:** Tongyao Yu, Haihong Zhou

**Affiliations:** ^1^Orthopaedic Trauma Department of Wenling First People's Hospital, Wenling 317500, Zhejiang, China; ^2^Hand and Foot Surgery Department of Wenling First People's Hospital, Wenling 317500, Zhejiang, China

## Abstract

At present, the most commonly used surgical treatment for fractures caused by external force injury is clinical, and unsupervised data mining is more advantageous in the face of the unknown format of perioperative network data. Therefore, this research aims to explore the application effect of unsupervised data mining in the concept of rapid rehabilitation nursing intervention after fracture surgery. 80 patients who underwent fracture surgery in the Department of Orthopedics of XXX Hospital were determined as the subjects, who were rolled into a research group (group R, 40 cases) and a control group (group C, 40 cases) by drawing lots. An unsupervised data mining algorithm based on unsupervised data mining for support vector machines (VDMSVMs) was proposed and applied to two groups of patients undergoing perioperative fracture surgery with the rapid rehabilitation nursing intervention and basic routine nursing. The results showed that the number of important features selected by the VDMSVM algorithm (5) was obviously more than that of the compressed edge fragment sampling (CEFS) algorithm (1) and the multicorrelation forward searching (MCFS) algorithm (2) (*P* < 0.05). The number of noise features screened by the VDMSVM algorithm (3) was much less in contrast to that of the CEFS algorithm and the MCFS algorithm, which was 8 and 10, respectively (*P* < 0.05). The Visual Analogue Scale (VAS) scores of the fracture site at the 4^th^, 8^th^, 12^th^, and 16^th^ hour after surgery in group R were all lower than the scores in group C (*P* < 0.05). The length of hospital stay (LoHS) in group R was greatly shorter than that in group C (*P* < 0.05). After different nursing methods, the World Health Organization Quality of Life (WHOQOL-BREF) score of patients in group R (89.64 points) was greatly higher than the score in group C (61.45 points) (*P* < 0.05). The nursing satisfaction score of group R was 92.35 ± 3.65 points, and that in group C was 2.14 ± 1.25 points, respectively (*P* < 0.05). The test results verified the effectiveness of the feature selection of the VDMSVM algorithm. The rapid rehabilitation nursing intervention was conductive to reducing the postoperative pain of fracture patients, shortening the LoHS of patients, improving the quality of life (QOL) of fracture surgery patients, and increasing the patient's satisfaction with nursing.

## 1. Introduction

Fracture refers to the interruption of the integrity of the bone. In most cases, the fracture is caused by external force stimulation, and most of the treatments used in clinical practice are surgical treatment [1–3]. The purpose of fracture surgery is to repair the basic shape of the relevant bone tissue to the greatest extent and rebuild the movement function and lever function of the skeleton. The functional rehabilitation of fracture patients requires early, active, and comprehensive nursing care [4, 5]. Traditional rehabilitation care is to let patients take long-term bed rest, but studies have pointed out that if patients stay in bed for too long after fracture surgery, it will lead to osteoporosis, tendon damage, and other conditions, so as to increase the pain. As a comprehensive nursing intervention, rapid rehabilitation nursing intervention is highly recognized by clinicians and fracture patients due to its own advantages. It can significantly alleviate the clinical symptoms of patients, decrease the number of hospital stays, and reduce the incidence of complications [6].

Feature selection is a key technology used in imaging evaluation. It maintains the recognition accuracy after removing irrelevant features on the basis of maintaining the original target features, and it can be applied to imaging evaluation after fracture [7, 8]. According to the types of network data, feature selection algorithms can be divided into semisupervised feature selection (SSFS), supervised feature selection (SFS), and unsupervised feature selection (UFS). Generally, SSFS or SFS is performed on the marked training data. However, in practical applications, the number of marks obtained is small, which has certain limitations [9, 10]. In UFS, feature selection can still be performed even for unlabeled data, and the entropy-based unsupervised data mining mode can automatically extract the combination of the largest amount of information from massive data, which is very suitable for highly discrete data. Perkins et al. [11] evaluated the fracture operation based on the unsupervised data mining under the *F*-sore, optimized the problem, achieved feature selection by solving the optimization problem, and targeted feature extraction. The algorithm must be run in the original feature set of manual marking, and the autonomous learning ability is seriously insufficient [12, 13]. In order to solve the above problems, an unsupervised data mining based on the unsupervised data mining for support vector machine (VDMSVM) algorithm was proposed in this study. The algorithm inputted raw data and did not require to manually construct candidate features before feature selection was performed and can filter the target features directly from the network data of unknown format. The rapid rehabilitation nursing intervention for fracture surgery patients during the perioperative period is effective and can effectively reduce the incidence of complications. In addition, the VDMSVM algorithm can select key features from the original network data, filter the unknown format network data, and connect the features to the model training, which greatly improves the performance of the algorithm.

In order to explore the rapid rehabilitation nursing intervention concept application in fracture surgery effect, the VDMSVM algorithm was proposed and applied to patients undergoing rapid rehabilitation nursing intervention and basic routine nursing fracture surgery perioperative patients so as to provide evidence for clinical nursing.

## 2. Research Objects and Their Grouping

80 patients who underwent fracture surgery in the Orthopedics Department of XXX Hospital from March 15, 2020, to May 23, 2021, were selected and rolled into a research group (group R, 40 cases) and a control group (group C, 40 cases) using the random lottery method, including 34 males and 46 females, with an average age of 61.2 ± 3.5 years. The study had been permitted by the Medical Ethics Committee, and the patients had understood it and signed the informed consent forms.

### 2.1. Inclusion Criteria

The inclusion criteria were determined as follows: patients who actively cooperated with the fracture surgery treatment; patients without abnormalities in other body organs except for the fracture site; and patients over 20 years old.

### 2.2. Exclusion Criteria

The exclusion criteria were given as follows: patients with severe neurological diseases and cognitive dysfunction, patients with coagulation dysfunction, and patients with liver and kidney dysfunction and peptic ulcer.

### 2.3. Treatment Methods

Subjects in both group R and group C were treated with surgery.

Patients in group C were performed with basic routine treatments. The specific procedures and precautions of the perioperative period were instructed before the surgery. Fasting was started 10 hours and drinking was forbidden 6 hours before the surgery. The routine surgical nursing and routine anesthesia were performed during the surgery. After the surgery, the patient was given routine infusion and common medication for analgesia. According to the actual situation, the patient was allowed to exercise the lower limb function independently, and the urinary catheter was removed 3 days after the surgery.

In group R, nursing staff communicated with the patient, informed the patient of the surgical procedure, possible conditions, and corresponding treatment measures before the surgery to relieve the patient's nervousness and panic, and improved the patient's cooperation. One day before the surgery, the patient's diet was mainly liquid food, rich in vitamins; 2 hours before the surgery, the patient was required to take functional beverages without special additives and started to refrain from drinking. During the surgery, nursing staff had to pay attention to the temperature and humidity in the operating room, take appropriate measures to keep warm, perform anesthesia with nerve block, and reduce the use of opioids. Nursing staff had to strictly control the patient's infusion volume after the operation and give analgesics 48 hours after the surgery. According to the patient's own situation, specific functional exercise measures should be formulated to ensure the patient's exercise volume. If the patient suffered from postoperative urinary retention, a urinary catheter should be inserted and removed 6 hours later.

### 2.4. Observation Indicators

The Visual Analogue Scale (VAS) of the fracture site of the two groups of patients was calculated at the 4^th^, 8^th^, 12^th^, and 16^th^ hour after surgery; and the length of hospital stay (LoHS) and the incidence of complications in the two groups were counted and compared. A self-made questionnaire survey was used to count patients' satisfaction with nursing. There were a total of 25 questions, each with a score of 1–4, including “dissatisfaction,” “satisfaction,” “general satisfaction,” and “very satisfaction” (100 points). The World Health Organization Quality of Life (WHOQOL-BREF) was adopted to assess the quality of life (QOL) of patients after surgery.

### 2.5. Construction of the VDMSVM

It was supposed that there were *N* network data {*X*_1_, *X*_2_, *X*_3_,…, *X*_*n*_}, *X*_*i*_ was a *q*-dimensional vector, and *X*_*i*_ (*I* = 1,…, *n*) was to represent the *i*th data, so its corresponding classification mark was denoted as *Y*_*i*_, and (*X*_*i*_, *Y*_*i*_) obeyed the probability distribution. A simple support vector machine (SVM) cannot accurately describe the features and cannot perform feature selection. The VDMSVM proposed in this study was to continuously optimize the following items:

(1) $$\begin{array}{c} \min A\overset{N}{\underset{i=1}{\sum }}\left[1-Y_{i}\left(X_{i}\alpha +\beta \right)\right]=\gamma \left\|\alpha \right\|+\frac{\delta {\left\|\alpha \right\|}_{2}^{2}}{2}. \end{array}$$

In equation (1), *A* represents a constant, *γ* and *δ* represent the adjustment parameters, the range of *Y*_*i*_ is [−1, 1], *α* represents a feature weight vector, *β* refers to an offset, and *N* refers to data volumes. On the basis of the supervised feature selection algorithm, the network data of unknown format are also unknown. At this time, they are transformed into an unsupervised feature selection:

(2) $$\begin{array}{c} \min A\overset{N}{\underset{i=1}{\sum }}B\left(Y_{i}f\left(X_{i}\right)\right)=\gamma \left\|\alpha \right\|+\;\frac{\delta }{2{\left\|\alpha \right\|}_{2}^{2}}. \end{array}$$

In equation (2), *B*( ) represents the loss function, *fX*_*i*_=*X*_*i*_*α*+*β*, *A* represents a constant, *γ* and *δ* represent the adjustment parameters, the range of *Y*_*i*_ is [−1, 1], *α* represents a feature weight vector, and *β* refers to an offset.

### 2.6. Experimental Design and Analysis

Compressed edge fragment sampling (CEFS) algorithm increases the space required for storing edge information and reduces the computational complexity of the reconstruction process. Multicorrelation forward searching (MCFS) algorithm optimizes lead sets and improves system performance. In order to verify the effectiveness of feature selection results of the VDMSVM algorithm, it was compared with the CEFS algorithm and the MCFS algorithm in this study. The *k*-means clustering (KMC) algorithm was adopted to test the selected feature subsets, the quality of the selected feature subsets was assessed according to the test results, and the effectiveness of the features was evaluated with the error of the final test. The performance of the VDMSVM algorithm was evaluated using the nonlinear dataset of the simulation experiment, and the final performance evaluation indicators obtained included the test error, the number of important features, the number of noise features, and the running time. In the simulation experiment, there were two kinds of data generated by the simulation, the data dimension *q* = 100, and the training data and the test data were both 2500. The parameters were set to the optimal solution which reached at 200 times of cross-validation.

### 2.7. Statistical Analysis

The data were analyzed and processed by SPSS 19.0. Measurement data were expressed by mean and standard deviation ($\bar{x}$ ± *s*), and *t*-test was performed. Counting data were expressed in percentage, and chi-square test was performed. The one-way analysis of variance (ANOVA) was for pairwise comparison. *P* < 0.05 indicated that there was a statistical difference.

## 3. Results and Discussion

### 3.1. Comparison Results on Performances of Three Algorithms

The performances of the three algorithms were compared for specific analysis, as illustrated in Figure 1. It illustrated that the test error of the VDMSVM algorithm (12.5%) was obviously lower than that of the CEFS algorithm (38.7%) and the MCFS algorithm (42.6%), showing a statistically great difference (*P* < 0.05). The number of important features screened by the VDMSVM algorithm (5) was more in contrast to the CEFS algorithm (1) and the MCFS algorithm (2), showing statistically visible differences (*P* < 0.05). In addition, the number of noise features selected by the VDMSVM algorithm (3) was obviously less than that of the CEFS algorithm (8) and the MCFS algorithm (10) (*P* < 0.05). However, while the VDMSVM algorithm showed good performance, its running time (9.5 s) was much longer than the CEFS and MCFS algorithms, which were 2.6 s and 3.1 s, respectively (*P* < 0.05). CEFS and MCFS algorithms' feature selection results were not very ideal, while VDMSVM algorithm was mainly for nonlinear data, and the feature selection effect was good. When raw network data were entered, the VDMSVM algorithm could automatically filter important features, while the CEFS and MCFS algorithms were relatively weak. Although VDMSVM algorithm could identify characteristic subsets with high capability, it took a long time, and its time cost needed to be reduced in the later period. In general, the VDMSVM algorithm could select key features from the original network data, perform feature screening on the unknown format network data, and integrate the features into the model training, which significantly improved the performance of the algorithm. The test results also showed the effectiveness of feature selection [14].

### 3.2. Comparison on General Data

The general data of the patients are compared, and the results are shown in Figure 2. Among them, there were 16 males and 24 females in group R, ranging in age from 58 to 65 years and 18 males and 22 females in group C, with an average age of 61.2 ± 3.5 years. The comparison results showed that no statistical difference could be found for general data of included subjects (*P* > 0.05).

### 3.3. Comparison of VAS Scores

The VAS scores of the fracture sites of the two groups of patients were calculated at the 4^th^, 8^th^, 12^th^, and 16^th^ hour after surgery, as shown in Figure 3. It revealed that the VAS scores were obviously lower in group R (4.5 points, 3.1 points, 2.3 points, and 1.2 points, respectively) than those in group C (5.9 points, 4.8 points, 4.5 points, and 3.9 points, respectively) at the 4^th^, 8^th^, 12^th^, and 16^th^ hour. All of the above values showed statistically remarkable differences (*P* < 0.05). Such results suggest that rapid rehabilitation nursing intervention is beneficial to relieve the postoperative pain and improve the prognosis of patients, which is consistent with the findings of Kim et al. [15].

### 3.4. Comparison on LoHS

Figure 4 shows the comparison results of the LoHS of patients in groups R and C. As it is given, the LoHS of group R (8.3 days) was greatly shorter than that of group C (13.5 days), which was statistically different (*P* < 0.05). This means that rapid rehabilitation nursing intervention can reduce the number of days in the hospital to a certain extent, thereby reducing the hospitalization costs and alleviating the economic pressure of patients. Such results matched to the conclusions of Segevall et al. [16].

### 3.5. Comparison on the WHOQOL-BREF Score

The WHOQOL-BREF scores of patients were compared, as illustrated in Figure 5. Before nursing, there was no statistical difference in the WHOQOL-BREF score between groups R and C (*P* > 0.05). After different nursing methods, the WHOQOL-BREF scores of the group R patients were greatly higher compared with the scores of group C, with statistical differences (89.64 points vs. 61.45 points; *P* < 0.05). This indicates that the rapid rehabilitation nursing intervention can improve the QOL of patients effectively treated with fracture surgery [17–19].

### 3.6. Comparison on the Incidence of Complications

Table 1 shows the postoperative complications of patients. The number of patients with incision infection, thrombosis, muscle atrophy, fat embolism, and shock was 1, 2, 1, 3, and 1 in the experimental group and 6, 8, 7, 9, and 5 in group C, respectively. The incidences of the above complications were statistically different between the two groups (*P* < 0.05). This discloses that the rapid rehabilitation nursing intervention for fracture surgery patients during the perioperative period is effective and can effectively reduce the incidence of complications [20].

### 3.7. Comparison on Nursing Satisfaction from Patients in Two Groups

The nursing satisfaction scores of patients were compared. The data in Table 2 showed that the nursing satisfaction score in group R was obviously higher than that of group C, which was 92.35 ± 3.65 points and 2.14 ± 1.25 points, respectively, with statistical differences (*P* < 0.05). This shows that rapid rehabilitation nursing intervention is unanimously recognized by patients, which can not only effectively relieve the nurse-patient relationship but also greatly improve the patient's satisfaction with the medical staff care [21, 22].

## 4. Conclusion

Based on the VDMSVM, the rapid rehabilitation nursing intervention was utilized to analyze the nursing effect of perioperative patients after fracture surgery. The test error of the VDMSVM algorithm was 12.5%, the number of important features was 5, and the number of noise features was 3. The test results verified the effectiveness of the feature selection of the VDMSVM algorithm. In addition, the rapid rehabilitation nursing intervention was conducive to relieving the postoperative pain of fracture patients, shortening the LoHS of the patients, improving the QOL of the patients undergoing fracture surgery, and increasing the satisfaction of the patients with nursing degree. The shortcoming of this study was that the sample size was small, which would interfere with the research results to a certain extent. In the later stage, the sample size has to be expanded for further in-depth exploration. In short, the rapid rehabilitation nursing intervention is currently in the preliminary stage of development, providing a new method for clinical fracture perioperative nursing.

## Figures and Tables

**Figure 1:** Comparison on the performance of three algorithms. (a–c) The comparison on the test error, numbers of important features and noise features, and running time, respectively. ^*∗*^The difference was statistically visible to the VDMSVM algorithm (*P* < 0.05).

**Figure 2:** Comparison on the general data of patients. (a, b) The comparison results of gender and age, respectively.

**Figure 3:** Comparison on VAS scores after fracture surgery. ^*∗*^An obvious difference statistically could be found (*P* < 0.05).

**Figure 4:** Comparison on LoHS for patients in two groups. ^*∗*^An obvious difference was visible (*P* < 0.05).

**Figure 5:** Comparison on the WHOQOL-BREF score for patients in different groups. ^*∗*^There was an obvious difference statistically (*P* < 0.05).

**Table 1:** Incidence of complications for patients.

	Research group	Control group	*χ* ^2^	*P*
Incision infection	1	6	6.358	<0.05
Thrombosis	2	8	9.267	<0.05
Muscle atrophy	1	7	10.354	<0.05
Fat embolism	3	9	11.261	<0.05
Shock	1	5	8.526	<0.05

**Table 2:** Comparison on the nursing satisfaction score.

Group	Number of patients	Nursing satisfaction score
Research group	40	92.35 ± 3.65 points
Control group	40	82.14 ± 1.25 points^*∗*^
*χ* ^2^	—	13.57
*P*	—	<0.05

^*∗*^The difference was statistically obvious (*P* < 0.05).

## Data Availability

The data underlying the results presented in this study are available within the article.

## References

[1] Gomez M., Rony L., Marc C. (2020). Fast-track care for pertrochanteric hip fracture: what impact on function and autonomy after discharge?. *Orthopaedics and Traumatology: Surgery & Research*.

[2] Pollmann C. T., Røtterud J. H., Gjertsen J.-E., Dahl F. A., Lenvik O., Årøen A. (2019). Fast track hip fracture care and mortality - an observational study of 2230 patients. *BMC Musculoskeletal Disorders*.

[3] Windsor T. A., Tewelde S. Z., Blosser K. M., Richardson A. C. (2020). An odontoid fracture and vertebral artery injury in fast‐track. *Clinical Case Reports*.

[4] Li H., Liu Y., Li Q., Fan J., Gan L., Wang Y. (2020). Effects of a fast track surgery nursing program in perioperative care of older patients with a hip fracture. *European Geriatric Medicine*.

[5] Kulshrestha V., Sood M., Kumar S., Sharma P., Yadav Y. K. (2019). Outcomes of fast-track multidisciplinary care of hip fractures in veterans: a geriatric hip fracture program report. *Clinical Orthopaedic Surgery*.

[6] Zhao H., You J., Peng Y., Feng Y. (2021). Machine learning algorithm using electronic chart-derived data to predict delirium after elderly hip fracture surgeries: a retrospective case-control study. *Frontiers in Surgery*.

[7] Moppett I. K., White S., Griffiths R., Buggy D. (2017). Tight intra-operative blood pressure control versus standard care for patients undergoing hip fracture repair - hip Fracture Intervention Study for Prevention of Hypotension (HIP-HOP) trial: study protocol for a randomised controlled trial. *Trials*.

[8] Gomez M., Marc C., Talha A. (2019). Fast track care for pertrochanteric hip fractures: how does it impact length of stay and complications?. *Orthopaedics and Traumatology: Surgery & Research*.

[9] Kohli S., Bawa A., Crooks S., Nagarajakumar A., Brooker J., Doddi S. (2019). A hip fracture nurse specialist has a positive outcome on the length of stay for patients with hip fractures. *Il Giornale di Chirurgia*.

[10] Nagano A., Maeda K., Shimizu A. (2020). Association of sarcopenic dysphagia with underlying sarcopenia following hip fracture surgery in older women. *Nutrients*.

[11] Perkins J. L., Perera S., Beach M., Esper S. A., Gruen G. S., Neft M. (2021). Probable delirium as a risk factor for adverse surgical outcomes in geriatric patients with acute hip fracture: preoperative assessment using a short screening tool. *AANA journal*.

[12] Wolfstadt J. I., Wayment L., Koyle M. A., Backstein D. J., Ward S. E. (2020). The development of a standardized pathway for outpatient Ambulatory fracture surgery. *Journal of Bone and Joint Surgery*.

[13] Hines C. B., Collins‐Yoder A. (2019). Bone cement implantation syndrome: key concepts for perioperative nurses. *AORN Journal*.

[14] Krupić F., Bišćević M., Spahić E. (2020). Experience of nurses in assessing postoperative pain in hip fracture patients suffering from dementia in nursing homes. *Medicinski Glasnik: Official Publication of the Medical Association of Zenica-Doboj Canton, Bosnia and Herzegovina*.

[15] Kim S.-J., Park H.-S., Lee D.-W., Lee J.-W. (2019). Short-term daily teriparatide improve postoperative functional outcome and fracture healing in unstable intertrochanteric fractures. *Injury*.

[16] Segevall C., Söderberg S., Björkman Randström K. (2019). The journey toward taking the day for granted again. *Orthopaedic Nursing*.

[17] Su S.-F., Lin S.-N., Chen C.-S. (2021). Self-efficacy care program for older adults receiving hip-fracture surgery. *Clinical Nursing Research*.

[18] Beaupre L. A., Moradi F., Khong H. (2020). Implementation of an in-patient hip fracture liaison services to improve initiation of osteoporosis medication use within 1-year of hip fracture: a population-based time series analysis using the RE-AIM framework. *Archives of Osteoporosis*.

[19] Krupic F., Grbic K., Senorski E., Lepara O., Fatahi N., Svantesson E. (2020). Experience of intensive care nurses in assessment of postoperative pain in patients with hip fracture and dementia. *Materia Socio Medica*.

[20] Parker M. J. (2017). Sliding hip screw versus intramedullary nail for trochanteric hip fractures; a randomised trial of 1000 patients with presentation of results related to fracture stability. *Injury*.

[21] Chow S. K.-H., Qin J.-h., Wong R. M.-Y. (2018). One-year mortality in displaced intracapsular hip fractures and associated risk: a report of Chinese-based fragility fracture registry. *Journal of Orthopaedic Surgery and Research*.

[22] Zhu W., Yan Y., Sun Y. (2021). Implementation of Enhanced Recovery after Surgery (ERAS) protocol for elderly patients receiving surgery for intertrochanteric fracture: a propensity score-matched analysis. *Journal of Orthopaedic Surgery and Research*.

